RETRACTED

# Melatonin Mediates Osteoblast Proliferation Through the STIM1/ORAI1 Pathway

**DOI:** 10.3389/fphar.2022.851663

**Published:** 2022-03-22

**Authors:** Lili Cao, Keda Yang, Wei Yuan, Siming Zhou, Rui Zhao, Shui Qiu

**Affiliations:** ^1^ Department of Medical Oncology, First Hospital of China Medical University, Shenyang, China; ^2^ Department of Orthopedics, First Hospital of China Medical University, Shenyang, China; ^3^ Minimally Invasive Orthopedic Surgery Ward, Shenyang Orthopedic Hospital, Shenyang, China

**Keywords:** osteoporosis, melatonin, postmenopausal women, STIM1, Ca^2+^

## Abstract

Based on the positive correlation between bone mineral density and melatonin levels in blood, this study confirmed that melatonin supplementation prevents postmenopausal osteoporosis. We further confirmed that melatonin promotes an increase in intracellular calcium concentrations through the STIM1/ORAI1 pathway, thereby inducing the proliferation of osteoblasts.

**Introduction:** Osteoporosis (OP) is a progressive, systemic bone disease that is one of the main causes of disability and death in elderly female patients. As an amine hormone produced by the human pineal gland, melatonin plays an important role in regulating bone metabolism. This study intends to investigate the relationship between melatonin levels in human blood and bone density and to suggest the efficacy of melatonin in treating osteoporosis by performing *in vivo* and *in vitro* experiments.

**Methods:** We used liquid chromatography-tandem mass spectrometry to determine the serum melatonin levels in postmenopausal women with osteoporosis and young women with a normal bone mass. The bone density, BV/TV, Tb.Th, Tb.Sp and other indicators of postmenopausal osteoporosis and mice with a normal bone mass were detected by measuring bone density and micro-CT. The intracellular calcium ion concentration was detected using fluorescence microscopy and a full-wavelength multifunctional microplate reader, and the expression of SOCE-related genes and STIM1/ORAI1 proteins was detected using PCR and WB.

**Results:** This study confirmed that bone density positively correlates with the melatonin level in human blood. In the animal model, melatonin supplementation reverses postmenopausal osteoporosis. We explored the internal mechanism of melatonin treatment of osteoporosis. Melatonin promotes an increase in intracellular calcium ion concentrations through the STIM1/ORAI1 pathway to induce osteoblast proliferation.

**Conclusions:** This study provides an important theoretical basis for the clinical application of melatonin in patients with osteoporosis and helps to optimize the diagnosis and treatment of postmenopausal osteoporosis.

RETRACTED

## Introduction

Osteoporosis (OP) is a progressive systemic bone disease (Kanis et al., 2019) that is characterized by a decreased bone mass and deterioration of bone microstructure, both of which will lead to an increased risk of brittle fracture, which is more common in postmenopausal women (Barron et al., 2020). OP complicated with brittle fracture often requires surgical treatment, and many human and financial resources are needed for treatment and nursing care. This condition may lead to paralysis or death after the operation, which will impose a heavy burden on the family and society (Rossi et al., 2018). At present, bisphosphonates, dinozumab and selective estrogen receptor modulators are used to prevent osteoporosis in postmenopausal women (Deeks, 2018; Barrionuevo et al., 2019; Yuan et al., 2019). However, these drugs do not stimulate bone formation and have a variety of side effects, such as a tumorigenic risk, accompanied by a high cost and poor patient compliance. Therefore, new drugs for the treatment of osteoporosis must be developed.

Melatonin is an amine hormone mainly produced by the pineal gland. It exists in many organisms, and its content changes over time (Zisapel, 2018). Melatonin is involved in regulating various processes in the human body, including blood pressure, core temperature, sleep, gastrointestinal physiology, anti-inflammatory function, and cardiovascular function (Xie et al., 2017; Yin et al., 2018; Zhong and Liu, 2018; Hardeland, 2019; Chitimus et al., 2020). Notably, postmenopausal women are prone to osteoporosis, and they often have a low melatonin level (Blaicher et al., 2000). Therefore, we speculate that melatonin may be closely related to the occurrence and development of osteoporosis. However, evidence of a clear correlation between melatonin levels and bone mineral density is lacking. As shown in previous research from our team, the effect of melatonin on osteoblast proliferation is concentration-dependent (Liu et al., 2011). When melatonin is present at low concentrations of 10 nM–100 μM, it can promote the proliferation, differentiation and mineralization of osteoblasts and inhibit the activation of osteoclasts (Zhao et al., 2020). With increasing melatonin concentrations greater than 1 mM, it inhibits osteogenic proliferation (Qiu et al., 2020). Therefore, we speculate that low concentrations of melatonin promote the proliferation of osteoblasts and treat osteoporosis, but the specific mechanism is unclear.

Peter et al. examined the human embryonic kidney 293 cell line and found that the endoplasmic reticulum STIM1 (stromal interaction molecules 1) protein is a signaling protein necessary to activate the calcium release-regulated calcium (SOC) channel on the membrane surface. Upon translocation to the cell membrane, it interacts with the cell membrane SOC channel component protein ORAIl and opens the SOC channel to induced Ca^2+^ release-activated Ca^2+^ influx (store operated Ca^2+^ entry, SOCE) (Stathopulos et al., 2013), and Ca^2+^ influx is one of the key factors promoting cell proliferation. Although SOCE has been detected in osteoblasts (Hu et al., 2014), the role of melatonin is unclear.

RETRACTED

This study aims to clarify the correlation between melatonin and bone mineral density and to further explore the mechanism by which melatonin promotes osteoblast proliferation through the STIM1/ORAI1 pathway to provide a theoretical basis for its use as a treatment for osteoporosis. This study provides a new entry point for the diagnosis and treatment of osteoporosis.

## Methods

### Recruitment and Enrollment

The study was approved by the Ethics Review Committee of the First Affiliated Hospital of China Medical University. We employed several recruitment methods, including distributing leaflets, advertising and using the internet. Women interested in participating in this research project called our special research phone number, and we interviewed the women who called. Potential participants were screened for eligibility through initial telephone interviews. The inclusion criteria included postmenopausal women aged 55–65 years and young women aged 20–25 years. If the preliminary inclusion criteria were met, the interview continued to ask about the exclusion criteria. The exclusion criteria included drugs currently being taken to treat osteoporosis or osteoporosis in the last three months, uncontrolled hypertension, hyperparathyroidism, liver and kidney diseases, diabetes, cancer, chronic obstructive pulmonary disease, and severe sleep apnea. Those who were considered eligible to participate were invited to arrange an initial visit to the orthopedic nursing center of the First Affiliated Hospital of China Medical University and a copy of the informed consent form containing information about the first visit and the research trial was provided to potential participants.

After participants who met the aforementioned conditions understood and expressed their desire to participate in the study and signed the informed consent form, we used dual energy X-ray (medi link) to screen and classify the participants’ bone health. Young women with T scores > - 1 and <1 were included in the normal group, and postmenopausal women with T scores < - 2.5 were included in the osteoporosis group.

### Collection and Storage of Serum Samples

Serum samples were collected bimonthly (morning at 6:00) (Melatonin secretion often peaked from 2 to 4 a.m., then gradually decreased and reached the lowest level at noon. Because our subjects were recruited and not hospitalized patients, we couldn’t get the serum samples from 2 to 4 a.m. We took the 6:00 a.m. period close to the peak to detect the serum melatonin level. At this time, the decline of serum melatonin level was low.) during daytime study appointments. Participants needed to fast overnight, and blood was obtained through venipuncture. The sample was incubated at room temperature for at least 30 min and then centrifuged at 4000 g for 10 min. The serum was taken collected the separated sample, divided equally and stored at −20°C until use.

RETRACTED

### Serum Melatonin Levels

The daytime serum melatonin level of each participant was measured in collected blood samples. Serum samples were analyzed using liquid chromatography-tandem mass spectrometry (SCIEX 6500, United States) according to the manufacturer’s instructions. A standard curve was generated for the assay according to the manufacturer’s instructions, and the melatonin level was calculated in pg/ml.

### Animal Model Construction and Experimental Design

Thirty 8-week-old female pathogen-free (SPF) C57B6 mice were purchased from the animal Department of China Medical University and housed in a metabolic cage on a 12 h light/12 h dark cycle for two weeks to adapt to the environment. The mice were randomly divided into three groups: sham operation group (*n* = 10), OVX group (*n* = 10), and OVX + melatonin group (60 mg/kg/d, *n* = 10. Melatonin was administered by gavage, and the body weights of the mice were recorded weekly for 8 weeks. Two months after modeling, the left femur and right femur were dissected from each group of mice. The Medical Ethics Committee of China Medical University approved the study.

### Measurement of BMD

Samples of mouse femurs were immersed in PBS at room temperature 2 months after melatonin treatment, and BMD was measured using dual energy X-ray absorptiometry (DCS-600R; Aloka, Tokyo, Japan) and reported as the bone mineral content per unit area.

### Bone Microstructure Observation

Mouse femoral samples were incubated in PBS at room temperature, and quantitative tomography was performed with micro-CT to analyze the microstructural parameters of cancellous bone, such as bone volume/total volume (BV/TV), bone trabecular number (Tb.N), bone trabecular thickness (Tb.Th), and bone trabecular separation (Tb.Sp).

### Cell Culture and Cell Viability Assay

Mouse osteoblast MC3T3-E1 cells were purchased from the cell bank of the Chinese Academy of Sciences (Shanghai, China), and cultured in *α*-MEM (Clone, Logan, Utah, United States) supplemented with 10% FBS (HyClone, Logan, Utah, United States) and 100 U/ml penicillin solution µg/ml streptomycin (HyClone, Utah, United States). The cultures were stored in a humidified incubator (Thermo Fisher Scientific, Massachusetts, United States) containing 5% CO_2_ at 37°C. The activity of melatonin-treated osteoblasts was determined using Cell Counting Kit 8 (Japan Tongren Molecular Technology Company). The absorbance of each well was measured at 450 nm using a microplate reader (Bio-Rad, Hercules, CA, United States) according to the manufacturer’s instructions. Cell viability was determined by calculating the mean absorbance of the melatonin treatment group/absorbance × 100% of the control group.

RETRACTED

### Reverse Transcription-Quantitative PCR Assay

Total RNA was extracted using the miRneasy RNA Mini Kit (Qiagen, MD, United States) according to the manufacturer’s instructions. Goscript™ Reverse transcription Mix Oligo (DT) (Promega, WI, United States) was used to synthesize cDNA templates. GoTaq^®^ QPCR Master Mix (Promega, WI, United States) was used for qPCR, and a Roche Light Cycler^®^ 480 II system (Roche, Basel, Switzerland) was used for data collection. The following PCR cycling program was used: 95°C for 2 min and 40 cycles of 95°C for 15 s and 60°C for 60 s. The sequences of all primers are shown in Table 1, and GAPDH was used as an internal control for normalization. Gene expression was calculated using the 2^−ΔΔCt^ method.

**TABLE 1:** Primers for real‐time polymerase chain reaction.

GAPDH AGG​TCG​GTG​TGA​ACG​GAT​TTG TGT​AGA​CCA​TGT​AGT​TGA​GGT​CA
STIM1 GGC​GTG​GAA​ATC​ATC​AGA​AGT TCA​GTA​CAG​TCC​CTG​TCA​TGG
ORAI1 GAT​CGG​CCA​GAG​TTA​CTC​CG TGG​GTA​GTC​ATG​GTC​TGT​GTC

### Detection of the Intracellular Calcium Concentration

MC3T3-E1 cells were cultured in a 6-well plate at a density of 2×10^5^ cells/well. The cells were cultured with or without 100 nM or 10 μM melatonin. After 24 h of culture, the supernatant was removed, and the cells were washed twice with PBS and then digested with 0.25% trypsin. Digestion was stopped by adding *α*-MEM supplemented with 10% FBS. The cells were suspended and centrifuged (1000 rpm for 5 min). The supernatant was removed, and the cells were washed twice with PBS and centrifuged again to obtain cell pellets. Subsequently, the cells were stained with 200 μL of Fluo-4/AM (Beyotime, Shanghai, China) (5 μmol/L) and then incubated at 37°C for 30 min. Finally, the cells were washed three times with PBS. The results were quantified using a full-wavelength multifunctional microplate reader at an excitation wavelength of 490 nm and an emission wavelength of 525 nm.

RETRACTED

### Western Blotting

Cells were incubated with radioimmunoprecipitation analysis (RIPA) buffer on ice for 30 min to produce whole-cell lysates. The protein fraction was centrifuged at 12,000 g for 15 min at 4°C, and the supernatant containing the total protein was collected. Then, SDS–PAGE gels were used to separate the proteins before transfer to polyvinylidene fluoride (PVDF) membranes. The membrane was blocked with 5% BSA for 2 h and then incubated with the primary antibody overnight at 4°C. After this incubation, the secondary antibody coupled with horseradish peroxidase was incubated with the membrane at 4°C for 2 h, and the blot was observed using an enhanced chemiluminescence (ECL) system (UVP Inc., CA, United States). The protein level was normalized to the corresponding glyceraldehyde 3-phosphate dehydrogenase (GAPDH) signal, and the optical density was quantified using ImageJ software (NIH, MD, United States).

### Cell Transfection

Synbio Tech (Suzhou, China) designed and synthesized specific siRNAs for stromal interacting molecule 1 (GenBank Accession No. NM 009287.5). The transfection and inhibition efficiency of the three siRNA sequences was tested. The inhibitory efficiency of stim1-si-3 was the highest (73.8%), and the dose was selected as 50 nM. The siRNA duplex was transfected into the cells using Lipofectamine 3000 reagent (Invitrogen) according to the manufacturer’s instructions. Forty-eight hours after siRNA transfection, the cells were used in experiments. The sequences of all primers are shown in Table 2, and GAPDH was used as an endogenous control.

**TABLE 2:** Three different nonoverlapping RNAi duplexes with the following sequences were obtained.

STIM1-si-1 GCGACUUCUGAAGAGUCUAdTdT UAGACUCUUCAGAAGUCGCdTdT
STIM1-si-2 GAAAGUGAUGAGUUCCUAAdTdT UUAGGAACUCAUCACUUUCdTdT
STIM1-si-3 GGAAGUCAUCAGAAGUGUAdTdT UACACUUCUGAUGACUUCCdTdT
NC UUCUCCGAACGUGUCACGUdTdT ACGUGACACGUUCGGAGAAdTdT

### Statistical Analysis

All experiments reported in this article were repeated at least three times. Statistical analyses were performed using SPSS. ANOVA followed by Tukey’s post hoc tests was used to identify statistically significant differences. *p* < 0.05 was considered statistically significant.

## Results

### Illustrates the Difference in Serum Melatonin Levels Between Postmenopausal Women with Osteoporosis and Young Women with a Normal Bone Mass

To clarify the relationship between melatonin level and bone mineral density, We screened 50 postmenopausal women with osteoporosis and 50 young women with a normal bone mass. After participants meeting the eligibility criteria understood the study, expressed a desire to participate and signed the informed consent form, we analyzed their serum samples using liquid chromatography-tandem mass spectrometry. Figure 1 shows the melatonin levels measured in postmenopausal women and young women at 6:00 a.m. A significantly lower serum melatonin level was detected in women with osteoporosis than in young women with a normal bone mass.

RETRACTED

**FIGURE 1:** Melatonin levels in women with osteoporosis decreased significantly. Blood samples were collected at 6:00 a.m. to determine the melatonin content in postmenopausal women with osteoporosis and young women with a normal bone mass using liquid chromatography-tandem mass spectrometry. Experiments were performed in triplicate, and data are shown as the means ± standard deviations. *p < 0.05 or **p < 0.01 compared with young women.

### Melatonin Reverses Osteoporosis in Postmenopausal Mice

Our study revealed a significantly reduced serum melatonin level in women with osteoporosis, indicating a clear correlation between the melatonin level and bone density. Therefore, we verified whether the administration of melatonin can reverse the decrease in bone mass in postmenopausal mice. By testing bone density, we found that the bone mass in postmenopausal mice was significantly reduced, while the loss of bone mass was significantly reversed in animals treated with 60 mg/kg/day melatonin (Figure 2A). The BV/TV, Tb.Th, and Tb.Sp indicators of mice were detected using micro-CT. The BV/TV and Tb.Th of postmenopausal mice were significantly reduced, and Tb.Sp was significantly increased. After the administration of melatonin, BV/TV and Tb.Th were significantly increased, and Tb.Sp was significantly decreased (Figure 2B). Based on these results, melatonin significantly reverses the decrease in bone mass after menopause.

**FIGURE 2:** Melatonin significantly reverses postmenopausal osteoporosis. **(A)** Bone mass was detected in the mouse femur by measuring bone density. **(B)** BV/TV, Tb.Th, Tb.Sp indicators in the mouse femur were analyzed using micro-CT. Experiments were performed in triplicate, and data are presented as the means ± standard deviations. *p < 0.05 or **p < 0.01 compared with control cells.

### Melatonin Promotes Osteoblast Proliferation by Increasing Intracellular Calcium Levels

We found that melatonin significantly reversed the reduction in postmenopausal bone mass. We detected the effect of melatonin on osteoblast proliferation using the CCK-8 assay to better understand its mechanism. In MC3T3-E1 cells treated with melatonin (10^−4^, 10^−5^, or 10^−6^ mM), 10^−5^ mM and 10^6^ mM melatonin promoted osteoblast proliferation, whereas 10^−4^ mM melatonin had no effect on osteoblast proliferation (Figure 3A). In addition, by detecting the intracellular calcium concentration, we found that melatonin significantly increased the intracellular calcium concentration (Figure 3B). Based on the effects of melatonin on osteoblasts, cells were treated with a TRPC calcium ion inhibitor, and the inhibitor significantly reduced cell proliferation (Figure 3C), indicating that melatonin induced osteoblast proliferation by increasing the intracellular calcium ion concentration.

RETRACTED

**FIGURE 3:** Melatonin induces osteoblast proliferation by increasing intracellular calcium concentrations. **(A)** Cells were treated with different concentrations of melatonin (0, 10^−4^, 10^−5^, or 10^−6^mM) for 48 h. Cell proliferation was detected by performing a cell viability test. **(B)** Cells were treated with melatonin (0, 10^−4^, 10^−5^, or 10^−6^ mM) for 48 h, and the fluorescence intensity of Ca^2+^ was examined using a full wavelength multifunctional microplate reader and fluorescence microscope. **(C)** The TRPC inhibitor was added, and cell proliferation was detected using a cell viability test. Experiments were performed in triplicate, and data are presented as the means ± standard deviations. *p < 0.05 or **p < 0.01 compared with control cells.

### Melatonin Induces Osteoblast Proliferation Through the STIM1/ORAI1 Pathway

We detected the expression of the SOCE-related genes STIM1 and ORAI1 using PCR to further explore the mechanism of melatonin-induced osteoblast proliferation (Figure 4A). The results showed that melatonin significantly upregulated the expression of the STIM1 and ORAI1 genes. In addition, we performed Western blotting to detect the expression of STIM1 and ORAI1 proteins (Figure 4B). Melatonin significantly upregulated the expression of STIM1 and ORAI1 proteins. We knocked out STIM1 in MC3T3-E1 cells to determine whether melatonin promotes osteoblast proliferation by upregulating STIM1 to increase the intracellular calcium concentration (Figure 4C). After STIM1 knockdown, the increase in intracellular calcium concentrations induced by melatonin was significantly reversed (Figure 4D). Therefore, melatonin induces an increase in the intracellular calcium ion concentration through the STIM1/Orai1 pathway, thereby promoting the proliferation of osteoblasts.

**FIGURE 4:** Melatonin induces osteoblast proliferation through the STIM1/ORAI1 pathway. **(A)** The expression of the SOCE-related genes STIM1 and ORAI1 was detected using PCR. **(B)** Levels of the STIM1 and ORAI1 proteins were detected using Western blotting. **(C)** Transfection efficiency of the STIM1 siRNA was determined by measuring mRNA and protein levels. **(D)** Fluorescence imaging and qualification of Ca^2+^ levels using the indicator dye Fluo-4 AM following STIM1-siRNA transfection.

RETRACTED

## Discussion

Osteoporosis is the most common disease characterized by abnormal bone metabolism in the elderly (Armas and Recker, 2012). With the accelerated aging of the population and changes in lifestyles, the high incidence of osteoporosis has not been effectively curbed and even shows an increasing trend worldwide (Lane, 2006). In our country, this situation is more prominent, and it is one of the main causes of disability and death in elderly female patients (Wang et al., 2009). Therefore, a thorough understanding of the mechanism underlying the occurrence and development of osteoporosis and precise and efficient diagnosis and treatment measures are the long-term research focus currently and in the future.

Mammalian pineal gland is the main source of melatonin in the blood. In the cerebrospinal fluid of the third ventricle of the brain, it helps to regulate the circadian rhythm system (Reiter, 1991). Melatonin is also synthesized in many external parts of the pineal gland, such as the brain, retina, lens, cochlea, immune system, lung, gastrointestinal tract, liver, kidney, thyroid, pancreas, thymus, spleen, carotid body, reproductive tract, and skin (Slominski et al., 2008; Hardeland et al., 2011; Acuña-Castroviejo et al., 2014). Most of the cells have the capacity to synthesize melatonin including bone marrow and osteoblast, mitochondria are the birth place, battle ground and the site of melatonin metabolism in cells (Reiter et al., 2018). Melatonin, as an amine hormone, plays an important role in regulating bone metabolism (Li et al., 2019). Studies have found that postmenopausal women have a higher probability of suffering from osteoporosis (Watts, 2018).

This may be closely related to the massive loss of estrogen in postmenopausal women (Li and Wang, 2018). Interestingly, melatonin levels in postmenopausal women tend to be lower (Toffol et al., 2014), but the relationship between melatonin levels and bone density is currently unclear. Our research have found that the level of melatonin in postmenopausal women with osteoporosis is significantly lower than that in young women with a normal bone mass, indicating that the level of melatonin is closely related to osteoporosis which can provide a theoretical basis for melatonin as an auxiliary diagnostic index of osteoporosis in the future. We confirmed that melatonin deficiency is closely related to bone loss, so whether melatonin supplementation can prevent the occurrence and development of postmenopausal osteoporosis. We treated postmenopausal mice with 60 mg/kg/day melatonin and measured the bone mineral density and BV/TV, Tb.Th, Tb.Sp and other indicators. The results show that melatonin supplementation can significantly prevent the progression of postmenopausal osteoporosis, but its mechanism is not clear.

RETRACTED

Previous studies have found that as an important factor regulating the normal physiological functions of cells (Cha and Noma, 2012), Ca^2+^ exerts an important regulatory effect on cell proliferation (Borowiec et al., 2014). Store-operated Ca^2+^ entry (SOCE) is the main pathway of Ca^2+^ influx (Prevarskaya et al., 2011), and it participates in regulating the proliferation of various cell types by modulating the expression of SOCE-related proteins (Ogata et al., 1991; Bootman et al., 2001; Capiod, 2011). SOCE is activated by the complex interaction between the Ca^2+^ channel protein ORAI1 on the cell membrane and the Ca^2+^ sensor protein STIM1 located in the endoplasmic reticulum, increasing the intracellular calcium ion concentration (Secondo et al., 2019; Yeung et al., 2020). Our research revealed that melatonin significantly increased the proliferation of osteoblasts. The intracellular calcium ion concentration was detected by fluorescence microscopy and a fluorescence microplate reader and found that melatonin significantly increased the intracellular calcium ion concentration. At the same time, we added the calcium ion inhibitor TRPC and found that osteoblast proliferation was significantly inhibited. This suggests that melatonin induces the proliferation of osteoblasts by promoting the increase of intracellular calcium ions. Next, We detected the expression of the STIM1 and ORAI1 proteins and found that melatonin significantly upregulated the expression of the STIM1 and ORAI1 mRNAs and proteins. Upon STIM1 knockout, the increased calcium ion concentration in the cells was significantly reduced. Thus, melatonin promotes an increase in intracellular calcium ion concentrations through the STIM1/ORAI1 pathway, thereby inducing osteoblast proliferation.

In summary, our study is the first to confirmed that bone density positively correlates with the level of melatonin in human blood. We also explored melatonin as a treatment for osteoporosis and deeply explore its internal mechanism. These results provide an important theoretical basis for the application of melatonin in patients with osteoporosis, actively promote the clinical application of melatonin, and help optimize the diagnosis and treatment of postmenopausal osteoporosis.

## Data Availability

The original contributions presented in the study are included in the article/Supplementary Material, further inquiries can be directed to the corresponding author.
